# ZNF354C Mediated by DNMT1 Ameliorates Lung Ischemia-Reperfusion Oxidative Stress Injury by Reducing TFPI Promoter Methylation to Upregulate TFPI

**DOI:** 10.1155/2022/7288729

**Published:** 2022-07-19

**Authors:** Qi Shi, Nana Feng, Qingyun Ma, Shaohua Wang, Huijun Zhang, Dayu Huang, Jiayuan Sun, Meng Shi

**Affiliations:** ^1^Department of Thoracic and Cardiovascular Surgery, Huashan Hospital, Affiliated with Fudan University, Shanghai 200040, China; ^2^Department of Respiratory Endoscopy, Department of Respiratory and Critical Care Medicine, Shanghai Chest Hospital, Shanghai Jiao Tong University, Shanghai 200030, China; ^3^Department of Respiratory and Critical Medicine, Shanghai Eighth People's Hospital Affiliated to Jiang Su University, Shanghai 200030, China

## Abstract

**Background:**

Pulmonary ischemia reperfusion- (I/R-) induced dysfunction is a significant clinical problem after lung transplantation. In this study, we aim to explore the molecular mechanism of lung I/R injury (LIRI).

**Methods:**

Bioinformatic analysis of gene involved in oxidative stress. A HUVEC oxygen glucose deprivation/reoxygenation (OGD/R) model and I/R mouse model were first established via I/R. The cellular proliferation, migration, reactive oxygen species (ROS), and parameters of lung injury were assessed via CCK-8, EdU staining, Transwell, cellular ROS kit, and H&E staining. We also confirmed related gene expressions and protein levels and the interaction between the tissue factor pathway inhibitor (TFPI) promotor and ZNF354C.

**Results:**

Bioinformatic analysis results showed TFPI contributed to oxidative stress. OGD/R caused a reduction in cell viability and migration, hypermethylation of TFPI, increased ROS, and downregulation of ZNF354C, TFPI, and DNA methyltransferases (DNMTs) in HUVECs. Besides, ZNF354C could directly bind to the TFPI promoter, enhance proliferation and migration, and inhibit ROS in OGD/R-induced HUVECs by upregulating TFPI. More importantly, we discovered that 5-Aza could reduce TFPI methylation, upregulate TFPI, and enhance the binding of ZNF354C to the TFPI promoter in LIRI. Furthermore, DNMT1 silencing could induce proliferation and migration and prevent ROS in OGD/R-induced HUVECs by upregulating ZNF354C. Additionally, we verified that ZNF354C could alleviate LIRI by preventing DNA methylation *in vivo*.

**Conclusions:**

ZNF354C overexpression induced proliferation and migration, as well as suppressed ROS in OGD/R-induced HUVECs, and alleviated LIRI in mice by inhibiting TFPI promoter methylation to upregulate TFPI. Therefore, ZNF354C and TFPI methylation might be promising molecular markers for LIRI therapy.

## 1. Background

During lung transplantation, acute lung injury (ALI) caused by the insufficient blood supply to the lungs and subsequent perfusion (denoted ischemia-reperfusion (I/R) injury [1] and “LIRI” when specific to the lung) [2] remain a challenging clinical problem, resulting in the high mortality after lung transplantation [3]. The success rate of lung transplantation is furthermore limited by high rates of primary graft dysfunction (PGD) [4]. LIRI is usually associated with acute, aseptic inflammation, alveolar damage, and vascular permeability [5, 6]. Furthermore, LIRI is also a complex pathophysiological process, which may be associated with neutrophil infiltration, endothelial cell injury, apoptosis, and necrosis [7, 8]. There are no therapeutic agents clinically utilized to specifically prevent LIRI, with treatment strategies limited to supportive care. Therefore, it is imperative to find effective molecular targets for LIRI therapy.

A tissue factor pathway inhibitor (TFPI), a multidomain and a Kunitz-type protease inhibitor of factor VIIa/tissue factor (TF), is produced primarily by endothelial cells and released after cellular stimulation [9]. Endothelial cells are one of the primary cell types for TFPI synthesis, and the endothelial-bound TFPI contributes to the antithrombotic potential of vascular endothelial cells [10]. Research verified that TFPI can increase the occurrence of autoimmune injury by promoting the overactivation of autoimmune factors or chemokines [11]. Moreover, the elevated TFPI level in sepsis may represent endothelial dysfunction [12]. TFPI also plays a key role in the regulation and function of endothelial permeability, which is associated with the development of sepsis and ALI [13]. Research has also shown that intratracheal TFPI can improve gas exchanges and prevent mortality in ALI model rats that presents with severe sepsis [14]. Importantly, endothelial-specific destruction of TFPI can enhance lung endothelial permeability and promote metastasis in lung metastatic tumor models. TFPI deficiency in endothelial cells also induces pulmonary tumor metastasis with increased vascular permeability and altered lung microenvironment [15]. Despite accumulating research into the effects of TFPI in ALI, the function and mechanism of TFPI in LIRI have not been elucidated.

Zinc finger proteins (ZNF) are a class of transcription factors with multiple functions [16]. Specifically, ZNF354C has been found to have a critical role in bone and tumors [17, 18]. To further investigate the possible mechanisms of TFPI in LIRI, we applied bioinformatic analysis to predict the potential proteins that can bind to the TFPI promoter and concluded that ZNF354C may have a direct targeting regulatory role with the TFPI promoter. We also found that ZNF354C was downregulated in oxygen-glucose deprivation/reperfusion- (OGD/R-) induced human umbilical vein endothelial cells (HUVECs). Therefore, we speculated that ZNF354C may regulate TFPI expression by targeted binding, thus affecting the developmental process of ALI. However, the regulatory mechanism of ZNF354C has not been reported yet.

Epigenetic modifications are reportedly to play a key role in disease progression and are widely involved in biological processes covering cell development, cycle, oxidative stress, and inflammatory responses [19]. Among the processes, DNA methylation is the most intensively studied epigenetic modification, which relies on the catalytic action of DNA methyl transferases (DNMTs) [20]. Therefore, DNMTs are key factors in regulating the methylation levels of target genes. DNA methylation is mainly regulated by three DNMTs, DNMT1, DNMT3a, and DNMT3b [21]. DNMT1 is considered the key enzyme for maintaining normal DNA methylation due to its high affinity for hemimethylated DNA duplexes [22]. Vast evidence suggests that DNMT1 can regulate cell cycle and tumor suppressor gene expression, which is crucial in tumor metastasis and linked to poor prognosis [23, 24]. Besides, studies have confirmed that DNMT1 is associated with other common diseases, such as type II diabetes [25], Alzheimer's disease [26], and periodontal disease [27]. Recent research also revealed that DNMT1 can mediate the polarization of M1 alveolar macrophages in ALI [28]. Lastly, our preliminary experiment also discovered that DNMT1, DMNT3A, and DMNT3B were memorably upregulated in OGD/R-induced HUVECs. However, the regulatory role between subtypes A and B is not clear.

In the present study, we established an *in vitro* and an *in vivo* I/R model to determine the effects of TFPI on LIRI. We discovered that TFPI was methylated under OGD/R condition in HUVECs. Besides, we further disclosed a protective role of TFPI in OGD/R HUVECs and I/R model mice. More importantly, we found that as a binding partner of TFPI, ZNF354C also could attenuate cell proliferation and migration of OGD/R-induced HUVECs via repressing the methylation of TFPI. These findings suggested that the ZNF354C/TFPI axis might be a potential therapeutic target for LIRI.

## 2. Methods

### 2.1. Microarray Data Download and Processing

We downloaded four different types of stem cells from geo database (https://www.ncbi.nlm.nih.gov/geo/query/acc.cgi?acc=GSE127003), including 46 pairs of expression data from peripheral human lung biopsies at the end of cold ischemia and after two hours of reperfusion following transplantation. We extracted the original data with R software package affyio, standardized the data with R software package oligo, and mapped the probe to the gene, When multiple probes are matched to a gene, take the median as the expression level of the gene, remove the multiple matched probes, and conduct single sample gene set enrichment analysis on each sample with R software package GSVA to obtain the enrichment fraction of each sample in different go biological processes. R software package pheatmap is used for heat map visualization.

### 2.2. Cell Culture and Treatment

HUVECs were purchased from ATCC (CRL-1730) and cultured in Dulbecco's modified Eagle's medium (DMEM; Gibco, Billings, MT, USA) supplemented with 10% fetal bovine serum (FBS, Gibco) in a humidified incubator with 5% CO_2_ at 37°C. For OGD/R treatment, HUVECs were incubated with glucose-free media in a closed tank with 95% N_2_ and 5% CO_2_ (replace the gas in the closed tank with 95% N2-5% CO_2_ (5 L/min flow rate for 15 min), so that the O_2_ content in the closed tank is less than 1%.) at 37°C for 4 h. Then, after replacing with conventional culture medium, cells were incubated in a 37°C, 5% CO_2_-95% O_2_ incubator for 3 h [29]. Cells were then changed to complete media and cultured for 6, 12, 24, 48, or 72 h, respectively, to perform subsequent assays.

### 2.3. Cell Transfection

Control short-hairpin RNAs (shRNAs) (shCTRL), DNMT1 shRNAs (shDNMT1), or ZNF354C shRNAs (sh ZNF354C) were gained from GenePharm (Shanghai, China). The sequence of DNMT1 shRNA was 5′-UGUUAAGCUGUCUCUUUCCAAdTdT-3′. The sequence of ZNF354C shRNA was 5′-AAAUGUAUAAUACAUAUUGGGdTdT-3′. HUVECs were cultured in a 6-well plate (2 × 10^5^ cells/well) and transfected with Lipofectamine 2000 based on the manufacturer's instruction. Vector control (OE-CTRL), ZNF354C overexpression plasmids, or DNMT overexpression plasmids were provided by HanBio Biotechnology (Shanghai, China). HUVECs were then transfected with 50 *μ*L lentivirus (10^7^ IU/mL), which were filtered with 6 *μ*g/mL polybrene. Then, cells were incubated for 48 h and collected for further study.

### 2.4. Cell Counting Kit-8 (CCK-8)

HUVECs under OGD/R (1 × 10^4^ cells/well) were seeded onto 96-well plate and transfected with the indicated plasmids. After 24, 48, and 72 h, 10 *μ*L of CCK-8 was added to HUVECs in each well. After 2 h, the absorbance of 450 nm was measured using by a microplate reader (Infinite M200, Tecan, Männedorf, Switzerland). Data are representatives of three independent experiments.

### 2.5. EdU Staining

The transfected HUVECs (2 × 10^5^ cells/well) were seeded onto a 12-well plate. Then, the EdU solution (10 *μ*M) was added to the cells and incubated for 2 h. Cells were fixed by 4% paraformaldehyde for 15 min, disposed of glycine (50 *μ*L), and permeabilized by 0.5% Triton X-100 for 15 min. FITC-labeled EdU was added to cells and further incubated for 30 min. Diaminophenylindane (DAPI) was utilized to label the nuclear. Images were taken by using a fluorescence microscope (Olympus IX73, Olympus Corporation, Tokyo, Japan).

### 2.6. Transwell Assay

The processed HUVECs in 6-well plate were digested using typsin and harvested. Then, HUVECs (1 × 10^5^ cells) were supplemented into the upper chamber of the transwell plate, and a total of 500 *μ*L complete medium was positioned into the lower chamber. After 24 h, HUVECs were stained with crystal violet and images were taken by a light microscope (Olympus BX41; Olympus Optical Co. Ltd., Japan). Four images were taken for each condition.

### 2.7. Would Healing

The processed HUVECs (1 × 10^5^ cells/well) in 12-well plates were incubated and adhered to the wall at 37°C. Then, an artificial gap was generated on the cell monolayer by a 200 *μ*L tip, and pictures were taken. After 24 h, the cell movement was tracked via light microscopy. The distance of cell movement was calculated.

### 2.8. RNA Extraction and Reverse Transcription Polymerase Chain Reaction (RT-qPCR)

Total RNA was extracted from the HUVECs or tissues by TRIzol reagent (Invitrogen, Carlsbad, CA, USA) according to the instruction of manufacturer. The first-strand cDNA was synthesized using a Bestar qPCR RT kit (DBI® Bioscience, Ludwigshafen, Germany). TFPI and ZNF354C were amplified by SYBR-Green PCR Master Mix (Applied Biosystems, Weiterstadt, Germany). The PCR procedure was 95°C for 2 min, followed by 95°C for 20 sec and 65°C for 1 min, total of 40 cycles. The primer sequences were as follows: GAPDH-F: 5′ TGTTCGTCATGGGTGTGAAC 3′ and GAPFH-R: 5′ ATGGCATGGACTGTGGTCAT 3′, TFPI-F: 5′ AGTTGCCACCACTGAAACT 3′ and TFPI-R: 5′ TCGCACTGTCGAGTGAAAAT 3′, ZNF354C-F: 5′ AAGTCCCTTCAGATACCCGT 3′ and ZNF354C-R: 5′ TGTCCCAGTGACCATCCTTA 3′. GAPDH was used as a negative control. The relative expression was calculated via the 2-^*ΔΔ*Ct^ method.

### 2.9. Western Blot

The processed HUVECs or lung tissues were lysed by radioimmunoprecipitation assay (RIPA; Sigma-Aldrich, St. Louis, MO, USA) buffer containing protease inhibitor. The protein concentration was determined by a bicinchoninic acid (BCA) protein assay kit. A total of 30-40 *μ*g protein was separated using 12% SDS-PAGE and transferred to polyvinylidene fluoride (PVDF; Beyotime, Shanghai, China) membrane. After blocking with 5% nonfat milk at room temperature for 1 h, membranes were incubated with the first antibodies (anti-TFPI antibody, anti-ZNF354C antibody, anti-GAPDH antibody, and anti-DNMT1 antibody) at 4°C overnight. The next day, membranes were washed with 1XTBST for three times and incubated with secondary antibodies for 1 h at room temperature. The results were visualized using ECL and the quantified by ImageJ software (ImageJ 1.32 J, National Institutes of Health, Bethesda, MD, USA).

### 2.10. Immunofluorescence

Following a previous study [30], the processed HUVECs were seeded onto polylysine-coated slides in 24-well plate. After 48 h, cells were fixed with 4% paraformaldehyde and permeabilized by 0.1% Triton X100. Cells were then blocked with 1% bovine serum albumin (BSA) in 1X phosphate-buffered saline (PBS) at room temperature for 30 min followed by incubating with TFPI antibody at 4°C overnight. The next day, cells were washed with PBS for three times and incubated with a secondary antibody for 1 h at room temperature. The nuclear was stained by DAPI. The images were taken with a fluorescence microscope.

### 2.11. Methylation-Specific Polymerase Chain Reaction (MS-PCR)

A standard phenol-chloroform protocol was used to extract the genomic DNA from the cultured cells. DNA was treated with sodium bisulfite using an EpiTect Bisulfite kit (Qiagen, Hilden, Germany), and PCR amplification was performed. The PCR reaction condition was as follows: predenatured at 95°C for 10 min, followed by 35 cycles of 95°C for 30 s, 56°C for 30 s, and 72°C for 30 s, and with a final extension at 72°C for 5 min. The primer sequences used for methylation analysis of TFPI were 5′ ATAATGGGCGGTTAGGTAGAGAC 3′ and 5′ CCTAAAATACCGAAATTACAAACGA 3′. The primer sequence set used for unmethylation analysis of TFPI was 5′ TAATGGGTGGTTAGGTAGAGATGA 3′ and 5′ CTAAAATACCAAAATTACAAACAAA 3′. The PCR products were separated by electrophoresis on the 2% agarose gel.

### 2.12. Chromatin Immunoprecipitation (ChIP) Assay

By referring to a previous study [31], HUVECs were cross-linked by adding formaldehyde at a final concentration of 1% and incubated at room temperature for 10 min. A final concentration of 125 mM glycine was added to cells to stop the cross-linking. Cells were then washed with ice-cold PBS and scraped off in a solution of PBS plus protease inhibitors and centrifuged at 1000 rpm for 4 min. Cell pellets were resuspended in lysis buffer and incubated for 10 min on ice. Nuclei were collected by centrifugation and resuspended in nuclear lysis buffer and sonicated to an average length of 300-600 bp. The supernatant was divided into two fractions: one was for control and the second was incubated with 5 *μ*g antibody at 4°C overnight with rotation. The next day, the immune complex was washed consecutively for 5 min with low-salt wash buffer, high-salt wash buffer, and LiCl wash buffer, respectively. Elution was reverse cross-linked by adding 0.3 M NaCl and incubated at 65°C for 1.5 h. DNA was collected and purified by QiaQuick spin columns, and 2 *μ*L of DNA was used for PCR reactions. The PCR primers were TFPI-1F: 5′ CCATTGAGCACTGAGTGAACC 3′ and TFPI-1R: 5′ CCTCCCTGCCTGATTCTCC 3′, TFPI-2F: 5′ CAGGGCATGAGGTAATAGGA 3′ and TFPI-2R: 5′ ATTTGGTGGTGACTGGAACA 3′, TFPI-3F: 5′ AAGCATTCTTTTTCAACTGATTACA 3′ and TFPI-3R: 5′ AGATCACTGGCAGTTGGGAAT 3′, RNA polymerase II-F: 5′ ATGCTGGGTCCTGCCTTAA 3′ and RNA polymerase II-R: 5′ ATGCCTCAGTTCCTTTGTTCC 3′.

### 2.13. Luciferase Assay

By referring to the relevant literature [32], HUVECs (0.8 × 10^4^ cells/well) were seeded onto a 24-well plate and transfected with TFPI wild-type (WT) or mutant plasmid (0.8 *μ*g/well) by Lipofectamine 2000. After 48 h of transfection, cells were washed twice with PBS and lysed by passive lysis buffer. Cell lysates were collected, and a 100 *μ*L LARII working solution was added and mixed. A total of 100 *μ*L Stop & Glo reagent was added and mixed, before the absorption was measured at 560 nm.

### 2.14. Electrophoretic Mobility Shift Assay (EMSA)

According to a previous reports [33], nuclear DNA was extracted by nuclear and cytoplasmic protein extraction kit (Beyotime, P0028). The reaction mixture contained nuclear protein, antibody, and either the probe or mutant probe and antibody. And the sequence of probe was 5′-CTGTTTCCTTCATCTGTTTCCTCCACTAAAAAAAAG-3′. After incubation for 20 min on ice, biotin labeled probe was added to the mixture and incubated for 10 min at room temperature. Non-denaturing TBE-polyacrylamide gel was used to resolve protein-DNA complexes from free DNA. After electrophoresis, the polyacrylamide gel was transferred PVDF membrane and cross-linked by ultraviolet exposure (254 nm, 20 min). The membrane was blocked and washed, and the results were determined by chemiluminescence detection.

### 2.15. Enzyme-Linked Immunosorbent Assay (ELISA)

Based on a previous study [34], HUVECs were lysed by RIPA buffer containing proteinase inhibitor on ice for 30 min to 2 h. The cell lysis or serum from mice was centrifuged at 12000 rpm for 10 min at 4°C. The MDA and TFPI content in the supernatant were determined by ELISA kit according to the manufacturer's instruction. The concentrations of MDA, nitric oxide synthase (NOS), and TFPI in bronchoalveolar lavage fluid (BALF) were quantified using ELISA kits (Elabscience Biotechnology, Wuhan, China) following the manufacturer's instructions. The absorption at OD_450_ was measured using a microplate reader.

### 2.16. ROS Detection

Following previous research [35], the level of reactive oxygen species (ROS) was analyzed using a DCFDA/H2DCFDA-Cellular ROS Assay (ab113851; Abcam, Cambridge, UK) according to the manufacturer's instruction.

### 2.17. Ischemia/Reperfusion Animal Model

As described in a previous study [36], total of 120 (6-8 weeks, male) mice were randomly divided into eight groups (five mice/group): control, I/R, I/R plus 5-Aza, I/R plus control lentivirus, I/R plus ZNF354C lentivirus, I/R plus control shRNA, I/R plus ZNF354C silencing, and I/R plus ZNF354C silencing and 5-Aza. For the I/R model, the mice were anesthetized by intraperitoneal injection of 50 mg/kg bodyweight pentobarbital sodium. After tracheotomy, mice were mechanically ventilated by tracheal intubation with a tidal volume of 0.6 ml, a ventilation rate of 120 breaths/min, an inspiration-to-expiration ratio of 1 : 2, and an inhalation oxygen concentration of 100%. The left chest was debrided, local skin was disinfected, and the 4th and 5th intercostal spaces were bluntly separated to fully expose the left hilum. The mice were injected with 5 U/g bodyweight heparin into the tail vein, and the left hilum was blocked with a vascular clamp at the end of expiration after 5 min, so that the left lung was ischemic for 90 min (the ischemic period). Then, the vascular clamp was removed, and the left lung was repercussed for 120 min (the reperfusion period). For 5-Aza treatment, 5-Aza was injected through the tail vein at a concentration of 1 mg/kg bodyweight. For lentivirus treatment, a total of 200 *μ*L virus (10^8^ pfu/mL) was injected through the tail vein. The mice were sacrificed 3 days after infection, and the left lung tissues were collected.

### 2.18. Lung Wet-To-Dry Ratio

After sacrifice, the wet left lung tissue was weighed, incubated at 60°C for 96 h, and weighed as dry weight [37]. These values were used to calculate the wet-to-dry ratios.

### 2.19. Evans Blue Staining

Evans Blue (1%, 2 mg/kg bodyweight, Sigma-Aldrich) was injected via the tail vein 2 h before sacrifice [38]. Then, the left lung tissue was weighed, homogenized, treated with formamide (100 mg/ml; Sigma-Aldrich, Shanghai, China), incubated at 37°C for 24 h, and centrifuged for 20 min at 10,000 g. The absorbance of the supernatant was measured at 620 nm, and the concentration of Evans Blue was calculated from the absorbance according to a standard curve.

### 2.20. FITC Dextran Assay

FITC dextran (1%, 200 *μ*L) was injected via the tail vein 2 h before sacrifice. The left lung tissue was weighed and homogenized. The fluorescence intensity was measured by the fluorescent microplate reader at an excitation of 485 nm and an emission of 538 nm. The FITC-conjugated dextran concentration was calculated with a standard curve.

### 2.21. Immunohistochemistry (IHC)

Lung tissue specimens were embedded in paraffin and sliced 4 *μ*m thick. The sections were dewaxed, rehydrated, immersed in 0.01 M citrate buffer (pH 6.0), and boiled in a pressure cooker for 15 min. The sections were blocked with 3% hydrogen peroxide for 10 min and then incubated overnight at 4°C with rabbit monoclonal antibody against TFPI (1 : 100). The sections were exposed to secondary antibody for 1 h at room temperature. The nuclear was stained by hematoxylin.

### 2.22. Haematoxylin and Eosin (H&E) Staining

Lung tissue specimens were embedded, sliced, dewaxed, and rehydrated for the IHC assay. Slides were stained with hematoxylin solution for 10 sec and washed with tap water for 10 min. The sections were immersed in eosin staining solution for 30 sec and washed with tap water for 10 min. The sections were dehydrated in ascending alcohol concentrations and cleared with xylene.

### 2.23. Statistical Analysis

All data were analyzed using GraphPad Prism v9.0. The data were presented as the mean ± standard deviation (SD). One- or two-way ANOVAs followed by Tukey's post hoc test were used to compare the results from multiple groups. *P* < 0.05 was considered statistically significantly different.

## 3. Results

### 3.1. TFPI Oxidative Stress

According to the 46 pair expression data from peripheral human lung biopsies at the end of cold ischemia and after two hours of reperfusion following transplantation, we found 19284 different genes. Compared with the differences of KEGG pathway between the two samples, the top 10 KEGG pathways with the most significant differences were observed, which mainly includes beta alanine metabolism, MAPK signaling pathway, circadian rhythm mammal, and peroxisome (Figure 1(a)). It was worth mentioning that peroxisome, beta alanine metabolism, and propanoate metabolism were significantly activated in end of cold ischemia samples, whereas p53, MAPK signaling pathway, and other pathways were significantly blocked (Figure 1(b)). In addition, lower activity of oxidative stress-related biological processes was observed in the end of cold ischemia samples (Figure 1(c)) and twelve of the 14 oxidative stress-related biological processes were significantly lower in the end of cold ischemia samples (Figure 1(d)). Furthermore, a tissue factor pathway inhibitor (TFPI) was found involved in response to oxidative stress. The role of TFPI in oxidative stress was further analyzed as follows.

### 3.2. Impacts of OGD/R on Cell Viability, Migration, DNMT, ROS, and TFPI in HUVECs

To confirm the possible mechanism and therapeutic method in LIRI, we first established the OGD/R cell model in HUVECs. CCK-8 signified that cell proliferation of HUVECs was notably reduced after 6 h of OGD/R and recovered with extended reoxygenation (Figure 2(a)). The EdU staining results also denoted that OGD/R diminished the proliferation of HUVECs, and with increasing reoxygenation time, cell proliferation was gradually increased (Figures 2(b) and 2(c)). Meanwhile, the transwell experiment showed lower cell migration in OGD/R-mediated HUVECs versus that in the control HUVECs, while cell migration was gradually increased with reperfusion time (Figures 2(d) and 2(e)). TFPI is mainly produced by endothelial cells and megakaryocytes [39, 40]. In this regard, we further found that ZNF354C was the predicted transcriptional factor of TFPI. It is known that ZNF354C is a transcriptional factor that can bind short DNA consensus motif [41, 42]. Next, we further investigated the expressions of key genes (TFPI and ZNF354C) in OGD/R treated HUVECs. The results showed that the expression and concentration of TFPI were memorably suppressed by OGD/R and then recovered with the extension time of re-oxygenation (Figures 2(f)–2(i)). We also discovered that OGD/R (6 h of reperfusion) could downregulate ZNF354C in HUVECs, which then could be reversed as the reperfusion time increases (Figures 2(f) and 2(i)). Besides, western blot displayed that DNA methyltransferase enzymes (DNMT1, DMNT3a, and DMNT3b) were memorably induced by OGD/R in HUVECs; then, the expressions of these proteins were gradually decreased with the increase of reperfusion time (Figure 2(i)). Likewise, we discovered that the level of ROS was also observably elevated in OGD/R-induced HUVECs; then, ROS level gradually decreased with the increase of reperfusion time (Figures 2(j) and 2(k)). Together, our data revealed that OGD/R could reduce cell viability and migration and increase ROS, which might be relevant to the functions of ZNF354C, TFPI, and DNMTs in HUVECs.

### 3.3. OGD/R Induced Hypermethylation of TFPI in HUVECs, and TFPI Could Interact with ZNF354C

Subsequently, we verified the regulatory relationship between DNA methylation, TFPI and ZNF354C. First, we discovered that OGD/R (6 h of reperfusion) could cause the hypermethylation of TFPI promoter in HUVECs, while the elevation of TFPI promoter methylation could be gradually decreased as the reperfusion time increases (Figures 3(a) and 3(b)). Second, we predicated the binding sites between TFPI and ZNF354C (Figure 3(c)). And the luciferase results indicated that ZNF354C overexpression raised the luciferase activity of the WT-TFPI promoter, while the luciferase activity of the Mut-TFPI promoter was not affected by ZNF354C overexpression in HUVECs (Figure 3(d)). The EMSA results showed that ZNF354C is bound directly to the promoter of TFPI (Figure 3(e)). The ChIP results signified that the level of TFPI promoter was notably lessened in the OGD/R (6 h of reperfusion) group versus that in the control group, which were also prominently restored in HUVECs with the extended perfusion time (Figure 3(f)). Similarly, ChIP results revealed that the association of RNA pol-II with TFPI was most abundant after 6 h of OGD/R in HUVECs (Figure 3(g)). In short, these data uncovered that TFPI was hypermethylated and could interact with ZNF354C in OGD/R-induced HUVECs.

### 3.4. ZNF354C Overexpression Induced Proliferation and Migration and Reduced ROS Level through Upregulating TFPI in OGD/R-Induced HUVECs

Next, we verified the underlying roles of ZNF354C and TFPI in the proliferation and migration of OGD/R-induced HUVECs. We first overexpressed and silenced ZNF354C in OGD/R-mediated HUVECs. The results showed that ZNF354C overexpression dramatically reversed the reduction of ZNF354C and TFPI expressions, whereas ZNF354C silencing prominently enhanced the downregulation of ZNF354C and TFPI expressions in OGD/R-mediated HUVECs (Figures 4(a) and 4(b)). Likewise, the results of ELISA and IF staining denoted that ZNF354C overexpression markedly upregulated TFPI and ZNF354C silencing prominently downregulated TFPI in OGD/R-treated HUVECs (Figures 4(c) and 4(d)). Besides, ZNF354C overexpression dramatically increased cell proliferation, which was inhibited by OGD/R in HUVECs; conversely, suppression of ZNF354C alleviated the reduction of cell proliferation caused by OGD/R in HUVECs (Figures 4(e), 4(f), and 4(h)). In addition, ZNF354C overexpression also observably reversed the cell migration, which was decreased by OGD/R, whereas ZNF354C silencing markedly promoted the reduction of cell migration caused by OGD/R (Figures 4(g) and 4(i)). The ZNF354C overexpression also markedly reduced the ROS level, which was increased by OGD/R, while ZNF354C silencing memorably promoted the ROS level caused by OGD/R (Figure S1A). Moreover, ChIP data revealed that the binding of ZNF354C to the TFPI promoter was memorably decreased by OGD/R treatment, which could also be recovered by ZNF354C overexpression or further reduced by ZNF354C silencing in HUVECs (Figure 4(j)). The binding of RNA pol II to UTR of TFPI was also prominently increased by ZNF3544 overexpression and decreased by ZNF354C silencing in HUVECs (Figure 4(k)). Overall, these findings certified that ZNF354C could enhance the proliferation and migration and decrease the ROS level of OGD/R-induced HUVECs by upregulating TFPI.

### 3.5. 5-Aza Decreased TFPI Methylation, Increased TFPI Expression, Accelerated Proliferation and Migration, Attenuated ROS Level, and Enhanced the Combination of TFPI and ZNF354C in OGD/R-Treated HUVECs

To further confirm whether the methylation of TFPI is involved in the regulation of cell proliferation and migration in HEVCs under OGD/R, we treated HUVECs with 5-Aza, an inhibitor of DNA methylation [43]. The MSP results indicated that elevated methylation level of the TFPI promoter could be notably attenuated by 5-Aza, especially high concentrations of 5-Aza, in OGD/R treated HUVECs (Figure 5(a)). Furthermore, the OGD/R-mediated decrease of TFPI expression could also be reversed by 5-Aza, especially high concentrations of 5-Aza, in HUVECs (Figures 5(b)–5(e)). In addition, we found that 5-Aza could also memorably recover the OGD/R-mediated reduction of cell proliferation and migration in HUVECs in a dose-dependent manner (Figures 5(f)–5(j)). Meanwhile, we also revealed that 5-Aza also could notably reverse the elevation of ROS level, which were caused by OGD/R in HUVECs with a dose dependent manner (Figure S1B). Moreover, ChIP results confirmed that OGD/R lowered the binding of the TFPI promoter and ZNF354C antibody in HUVECs, which could be recovered by 5-Aza (Figure 5(k)). The binding of ZNF354C and RNA polymerase II with the promoter of TFPI could be decreased by OGD/R, yet could be partially reversed by 5-Aza in HUVECs (Figure 5(l)). Thus, the results disclosed that 5-Aza could aggrandize the proliferation and migration of OGD/R-treated HUVECs by reducing TFPI methylation to increase TFPI expression.

### 3.6. DNMT1 Suppressed Proliferation and Migration, Increased ROS Levels, and Reduced the Interaction of TFPI and ZNF354C in OGD/R-Induced HUVECs

Next, we investigated the involvement of DNA methyltransferase (DNMT1) in cell proliferation and migration of OGD/R-induced HUVECs. The MSP results first displayed that the OGD/R-mediated increased methylation of the TFPI promoter could be further potentiated by DNMT1 overexpression, or reversed by DNMT1 silencing in HUVECs (Figure 6(a)). We also verified that the expression and concentration of TFPI were further decreased by DNMT1 overexpression and increased by DNMT1 silencing in OGD/R-mediated HUVECs (Figures 6(b)–6(e)). Overexpression and silencing of DNMT1 were also verified in western blotting results (Figure 6(c)). As exhibited by CCK-8 and EdU assays, overexpression of DNMT1 observably promoted the OGD/R-mediated inhibitory effects on cell proliferation, and knockdown of DNMT1 by shRNAs partly reversed the OGD/R-mediated inhibitory effects of OGD/R on cell proliferation in HUVECs (Figures 6(f), 6(h), and 6(i)). The results also signified that DNMT1 overexpression memorably enhanced the OGD/R-mediated inductive effects on ROS level, whereas DNMT1 knockdown notably weakened these effects on the ROS levels in HUVECs (Figure S1C). Meanwhile, OGD/R caused defects of cell migration that could be recovered by DNMT1 silencing, or contrastingly elevated by DNMT1 overexpression in HUVECs (Figures 6(g) and 6(j)). Furthermore, ChIP results uncovered that the binding of the ZNF354C antibody to the TFPI promoter could be markedly depressed by DNMT1 overexpression and heightened by DNMT1 knockdown in OGD/R-induced HUVECs (Figure 6(k)). The binding of ZNF354C and RNA polymerase II to the TFPI promoter was also weakened by DNMT1 overexpression and prominently facilitated by DNMT1 knockdown in OGD/R-induced HUVECs (Figure 6(l)). These results further indicated suppression of DNMT1 could partly reverse the OGD/R-mediated reduction in proliferation and migration of HUVECs.

### 3.7. Silencing of DNMT1 Accelerated Proliferation and Migration and Suppressed ROS Levels by Regulating ZNF354C to Target the TFPI Promoter in OGD/R-Induced HUVECs

Meanwhile, we tested whether the influences of DNMT1 on the progress of OGD/R-induced HUVECs are mediated by ZNF354C. Our results disclosed that TFPI could be memorably upregulated by DNMT1 silencing, while this upregulation in TFPI expression was blunted by ZNF354C silencing in OGD/R-induced HUVECs (Figures 7(a)–7(d)). We next discovered that cell proliferation and migration could be notably strengthened by DNMT1 silencing, while this enhancement could also be memorably reduced by ZNF354C silencing in OGD/R-induced HUVECs (Figures 7(e)–7(i)). Meanwhile, the results showed that the level of ROS could be lowered by DNMT1 silencing, while this reduction could be dramatically reversed by ZNF354C silencing in OGD/R-induced HUVECs (Figure S1D). Generally, our data verified that DNMT1 silencing could induce proliferation and migration of OGD/R-induced HUVECs through ZNF354C.

### 3.8. ZNF354C Alleviated LIRI by Suppressing DNA Methylation *In Vivo*

Furthermore, we also demonstrated the influence and mechanism of ZNF354C in a LIRI mouse model. The LIRI mouse model was constructed through ischemia for 90 min and reperfusion for 120 min. Afterwards, the mice were injected with ZNF354C overexpression plasmids, shZNF354C lentivirus, and 5-Aza. As displayed in Figure 7(a), the dry-to-wet ratio of lung tissues was notably enhanced in the I/R mice relative to that in sham mice, and the dry and wet ratio was also signally reduced by 5-Aza or ZNF354C overexpression in I/R mice, while ZNF354C silencing cancelled the protective effects of 5-Aza on lung injury (Figure 8(a)). Meanwhile, we adopted Evans Blue to assess the degree of cerebral thrombosis. And as verified in Figure 7(b), the content of Evans Blue was dramatically strengthened in the I/R group versus that in the sham group, and 5-Aza or ZNF354C overexpression could prominently reduce the content of Evans Blue in I/R mice, and ZNF354C silencing also could weaken the reduction of Evans Blue mediated by 5-Aza in I/R mice (Figure 8(b)). Evans Blue dye and FITC-Dextran which all could be adopted to evaluate the permeability of pulmonary microvasculature. We found that the changing trend of fluorescence intensity of FITC-Dextran was similar to that of Evans Blue in each group of mice (Figure 8(c)). H&E staining results revealed that in the control group, the pulmonary alveoli and interstitium were intact, and the alveolar septum showed uniform thickness without signs of alveolar wall thickening or inflammatory cell infiltration; in the I/R group, lung tissue was severely hyperemic and bleeding, with inflammatory cells; and degree of lung injury in 5-Aza or ZNF354C overexpression groups was lower than that of I/R group; inhibition of ZNF354C also aggravated I/R induced-lung injury mediated by 5-Aza (Figures 8(d) and 8(e)). Moreover, we proved that TFPI expression was markedly lowered in the I/R group versus that in the sham group, and 5-Aza or ZNF354C overexpression could prominently elevate TFPI level in I/R mice, while the elevation of TFPI expression mediated by 5-Aza also could be remarkably attenuated by ZNF354C silencing in the lung tissues of I/R mice (Figures 8(f), 8(g), 8(i), and S2). Similarly, ELISA data also signified that 5-Aza or ZNF354C overexpression prominently upregulated TFPI, and the upregulation of TFPI mediated by 5-Aza also could be reduced by ZNF354C silencing in the serum of I/R mice (Figures 8(f), 8(g), and 8(j)). Furthermore, results showed that the expression change of ZNF354C in each group was consistent with that of TFPI (Figures 8(g) and 8(h)). As I/R injury is directly related to the formation of reactive oxygen species (ROS), endothelial cell injury, increased vascular permeability, and the activation of neutrophils and platelets, cytokines, and the complement system. Our data certified that I/R induced prominent elevation of TFPI, MDA, and NOS levels in BALF, which could be prominently decreased by 5-Aza or ZNF354C overexpression; however, inhibition of ZNF354C again attenuated the decrease in the levels of TFPI, MDA and NOS in BALF (Figures 8(k)–8(m)). Consequently, our results indicate that 5-Aza or ZNF354C could play protective roles in lung LIRI, which is relevant to DNA methylation.

## 4. Discussion

Pulmonary I/R not only maintains lung vitality but also triggers a series of complex cascade reactions, collectively known as LIRI [44]. LIRI has been proved to induce postoperative morbidity in patients undergoing lung transplantation [7]. It is characterized by increased microvascular permeability, elevated pulmonary vascular resistance, pulmonary edema, and pulmonary hypertension [45]. Furthermore, it can cause prolonged mechanical ventilation and pulmonary hypertension, which can seriously affect the prognosis of patients [46]. Therefore, the prevention and mitigation of LIRI are of great practical significance. In our study, we first applied OGD/R to establish an *in vitro* I/R model in HUVECs. In addition, we also constructed an I/R mouse model to investigate the *in vivo* cellular mechanisms involved in LIRI development via genetic overexpression and RNA silencing of crucial genes (i.e., TFPI, ZNF354C, and DNMT1).

The pulmonary endothelial cells play crucial roles in the development of ALI by increasing pulmonary vascular permeability [47]. Endothelial cell apoptosis can also disrupt cell-cell and cell-extracellular matrix interactions and loss of endothelial barrier function, leading to direct or indirect ALI [48]. Furthermore, oxidative stress results from an imbalance in oxidative and antioxidant levels. In this regard, it has been shown that the “respiratory burst” caused by damaging factors can produce large amounts of ROS, which further aggravate lung injury [49]. In our study, we also discovered that OGD/R could suppress cell viability and migration and induce ROS production of HUVECs. A previous study found that during sepsis, lung-associated TFPI antigens, mRNA levels decreased, and TFPI activity suddenly decreased 2 h after bacterial infusion [50]. Tissue factor (TF) and TFPI levels in BALF supernatant are significantly higher in patients with idiopathic pulmonary fibrosis compared to healthy controls [51]. Overexpression of TFPI also results in improved hemodynamic performance and reduced pulmonary vascular remodeling in a murine model of hypoxia-induced pulmonary hypertension [52]. TFPI deficiency in endothelial cells has been linked to pulmonary tumor metastasis with an increased vascular permeability and altered lung microenvironment [15]. Knockdown of endothelial-specific TFPI exacerbates lipopolysaccharide (LPS) induced ALI via the NF-*κ*B signaling pathway [53]. Local administration of recombinant human TFPI attenuates both pulmonary and systemic coagulopathy. Furthermore, nebulized rh-TFPI modestly reduces the pulmonary inflammatory response and allows increased bacterial clearance in rats with direct lung injury caused by P. aeruginosa [54]. Therefore, TFPI may be a beneficial therapeutic agent in intravascular clotting, sepsis, cancer, and ALI to attenuate pathologic clotting. Our results also proved that the TFPI promoter could be highly methylated under OGD/R in HUVECs, whereas TFPI and DNMT were downregulated in OGD/R-induced HUVECs. Therefore, TFPI methylation might be of vital importance in LIRI.

The pathogenesis of tissue injury induced by I/R involves epigenetic regulation [55]. DNA methylation on CpG dinucleotides is applied to “shut down” gene expression in cells catalyzed by DNMTs [56]. DNA methylation plays a key role in I/R related organ damage, including kidney injury, cerebral ischemia, and ischemic heart disease [55]. In our study, we further certified that the methylation inhibitor (i.e., 5-Aza) could reverse the downregulation of TFPI in OGD/R-induced HUVECs by inhibiting TFPI promoter methylation. Besides, 5-Aza also induced proliferation and migration, as well as lowered ROS levels in the OGD/R-induced HUVECs. More importantly, 5-Aza reduced the TFPI methylation, upregulated TFPI, and enhanced the combination of TFPI and ZNF354C in LIRI.

In the ischemic brain, the expression of DNMT1 is upregulated in astrocytes [57]. Another study revealed that after 4 days of transient global cerebral ischemia, the expression of DNMT1 distinctively decreased in the ischemic CA1 region, which may be related to ischemia-induced delayed neuronal death [58]. In addition, the reduction, but not the absence of DNMT1 in post mitotic neurons, protects against ischemic brain injury [59]. However, the functional role of DNMT1 in pulmonary ischemia reperfusion has not been found. In our study, we also verified that DNMT1 was involved in the regulation of OGD/R in HUVECs. Furthermore, DNMT1 silencing accelerated proliferation and migration, as well as prevented ROS production in OGD/R-induced HUVECs, whereas DNMT overexpression aggravated the lung injury induced by OGD/R. Although the methylation of TFPI has not been proven in HUVECs or other cells, hypermethylation in the promoter region of TFPI-2 has been analyzed in various types of cancers, such as non-small cell lung cancer [60], esophageal carcinogenesis [61], gastric cancer [62], acute myeloid leukemia [63], glioblastomas [64], and cervical cancer [65]. Thus, we suggest that the TFPI promoter methylation is a major contributor to LIRI-induced damage.

Zinc finger proteins (ZNF) are a large group of transcription factors with differential functions [66]. A previous study reported that ZNF354C is a key transcriptional factor in carcinogenesis and the development of esophageal squamous cell carcinoma (ESCC) by regulating targets genes [67]. Recently, a study revealed that ZNF354C is expressed in vascular cells, while ZNF354C overexpression inhibits the endothelial sprouting by binding to specific endothelial relevant target gene promoter [18]. In our study, we also proved that ZNF354C, as a transcriptional factor, could directly bind the promoter of TFPI. And ZNF354C also could enhance the proliferation and migration and reduced the ROS level of OGD/R-induced HUVECs through TFPI. Moreover, DNMT1 silencing could accelerate the proliferation and migration, as well as suppress ROS production, of OGD/R-induced HUVECs by regulating ZNF354C. Therefore, we further uncovered the crucial effects of ZNF354C and TFPI methylation in LIRI.

Nevertheless, our study is not without limitations. First, DNMT1 was not involved in the *in vivo* experiments. Second, pulmonary fibrosis and angiogenesis were not explored. Third, the specific regulatory mechanism between ZNF354C and DNMT1 is not completely clear. Fourth, the roles and mechanisms of DNMT3a and DNMT3b in ALI have not been clarified. For future research, Evans Blue Staining should be replaced with Evans Blue-TTC staining.

## 5. Conclusions

Our study showed that ZNF354C could interact with TFPI, and upregulate TFPI by preventing TFPI promoter methylation in OGD/R-induced HUVECs. DNMT1 could also reduce the interaction of TFPI and ZNF354C (Figure 9). Functionally, we discovered that ZNF354C ameliorates LIRI by preventing TFPI methylation to upregulate TFPI. Therefore, our study verified the key roles of ZNF354C overexpression or inhibition in TFPI promoter methylation of LIRI. This research provides a theoretical basis for further understanding of the molecular mechanism of LIRI development, as well as an experimental basis for the clinical diagnosis and therapeutic biomarkers of patients with ALI.

## Figures and Tables

**Figure 1:** Bioinformatic analysis of gene expression in peripheral human lung biopsies at the end of cold ischemia and after two hours of reperfusion following transplantation. (a) The top 10 KEGG pathways with the most significant differences were observed. (b) Peroxisome, beta alanine metabolism, and propanoate metabolism were significantly activated in the end of cold ischemia samples, whereas p53, MAPK signaling pathway, and pathways were significantly blocked. (c) Lower activity of oxidative stress-related biological processes was observed in the end of cold ischemia samples. (d) Twelve of the 14 oxidative stress-related biological processes were significantly lower in the end of cold ischemia samples.

**Figure 2:** The impact of OGD/R on cell viability, migration, DNA methyltransferase, and TFPI in HUVECs. HUVECs were exposed to OGD for 4 h and reoxygenated for 6, 12, 24, 48, and 72 h. (a) Cell viability was tested by CCK-8. (b, c) HUVECs were subjected to EdU staining, and EdU-positive cells were calculated in each group. (d, e) Migrated cells were confirmed via Transwell, and five fields were summarized and counted. TFPI level was monitored with (f) RT-qPCR, (g) ELISA, and (h) IF in HUVECs after OGD/R. (i) Western blotting analysis of TFPI, ZNF345C, DNMT1, DMNT3a, and DMNT3b levels. (j) ROS level was tested using DCFDA/H2DCFDA-Cellular ROS Assay in each group. (k) Quantitative analysis of ROS relative fluorescence intensity. The experiments were repeated three times independently.

**Figure 3:** OGD/R induced hypermethylation of TFPI in HUVECs, and TFPI could interact with ZNF354C. (a) Methylation level of TFPI promoter was tested with MSP in OGD/R-treated HUVECs. (b) The methylation level was quantified based on MSP results. (c) The predicated binding sites between TFPI and ZNF354C. (d) Luciferase activity of TFPI promoter in ZNF354C-overexpressed HUVECs was determined by applying dual luciferase reporter gene. (e) EMSA was utilized to test the binding of TFPI promoter and ZNF354C. (f) The interaction between ZNF354C antibody and TFPI promoter was confirmed with ChIP in HUVECs under OGD/R. (g) HUVECs were incubated with Poly II antibody and beads, and the binding of RNA polymerase II on TFPI 5′UTR was examined using ChIP in HUVECs under OGD/R. The experiments were repeated three times independently.

**Figure 4:** ZNF354C overexpression induced proliferation and migration through upregulating TFPI in OGD/R-induced HUVECs. OGD/R-treated HUVECs were transfected with ZNF354C overexpression plasmids or shZNF354C, respectively. ZNF354C and TFPI expressions were assessed via (a) RT-qPCR and (b) western blot. (c) TFPI level was analyzed with ELISA kit. (d) IF staining of TFPI in the processed HUVECs. (e) Cell viability was evaluated by CCK-8. (f) HUVECs in each group were subjected to EdU staining. (g) The images of cell migration were obtained using Transwell. (h) EdU-positive cells were quantitated in line with EdU staining results. (i) Quantitative analysis of migratory cells. (j) The binding of ZNF354C and TFPI promoter was confirmed through ChIP in each group. (k) The binding of RNA polymerase II on TFPI 5′UTR was examined via ChIP. The experiments were repeated three times independently.

**Figure 5:** 5-Aza decreased TFPI methylation, increased TFPI expression, accelerated proliferation and migration, and enhanced the combination of TFPI and ZNF354C in OGD/R-treated HUVECs. OGD/R-mediated HUVECs were treated with 5-Aza (low: 0.1 *μ*M, mid: 1 *μ*M, high: 10 *μ*M) for 24 h. (a) MSP was utilized to identify the methylation level of TFPI promoter. TFPI level was certified by applying (b) RT-qPCR, (c) western blot, (d) ELISA, and (e) IF staining in the processed HUVECs. Cell proliferation was determined with (f) CCK-8 and (g) EdU staining. (i) Migration in HUVECs was tested with Transwell. (h) EdU-positive cells and (j) migrated cells were counted. (k) The impact of 5-Aza on the binding of ZNF354C and TFPI promoter was confirmed by ChIP. (l) ChIP was adopted to analyze the effect of 5-Aza on the binding of RNA polymerase II on TFPI 5′UTR. The experiments were repeated three times independently.

**Figure 6:** DNMT1 suppressed proliferation and migration and reduced the interaction of TFPI and ZNF354C in OGD/R-induced HUVECs. HUVECs under OGD/R were transfected with DNMT1 overexpression plasmids or shDNMT1, respectively. (a) MSP displayed the change in the methylation level of TFPI promoter. The level of TFPI was tested through (b) RT-qPCR and (c) western blot, (d) ELISA, and (e) IF staining. (f) EdU staining was utilized to confirm the change of proliferation. (g) Transwell exhibited the change of cell migration. (h) CCK-8 presented the change in cell viability. (i) Based on the EdU staining data, EdU-positive cells were quantitated. (j) Migratory cells were quantitated in line with Transwell data. (k) ChIP demonstrated the impact of DNMT1 on the binding of ZNF354C and TFPI promoter. (l) ChIP showed the influence of DNMT1 on the binding of RNA polymerase II on TFPI 5′UTR. The experiments were repeated three times independently.

**Figure 7:** Silencing of DNMT1 accelerated proliferation and migration by regulating ZNF354C to target TFPI in OGD/R-induced HUVECs. OGD/R-induced HUVECs were transfected with shDNMT1 or/and shZNF354C. TFPI expression was identified through (a) RT-qPCR and (b) western blot, (c) ELISA, and (d) IF staining. (e, h) The change of cell proliferation was confirmed with EdU staining, and EdU-positive cells were quantitated. (f, i) The change of cell migration was monitored with Transwell, and migratory cells were quantitated. (g) CCK-8 presented the change of cell viability. The experiments were repeated three times independently.

**Figure 8:** ZNF354C alleviated LIRI through suppressing DNA methylation *in vivo*. The I/R model was established and then was disposed of ZNF354C overexpression plasmids, shZNF354C lentivirus, and/or 5-Aza (each group contained 5 mice). (a) After sacrifice, wet and dry lung weights of mice were measured and compared with wet-to-dry ratios. (b) Evans Blue was injected via the jugular vein 1 h before sacrifice, and the absorbance of the supernatant was tested at 620 nm. (c) The fluorescence intensity of FITC-Dextran was confirmed with FITC dextran assay. (d) The pathologic structure of lung tissues was assessed by H&E staining. (e) The lung injury score was also calculated by ImageJ based on the H&E staining results. (f) The expression of TFPI was measured by IHC. (g) The expressions of ZNF354C and TFPI were identified by Western blot. (h, i) And ZNF354C and TFPI expressions were quantified. EILISA kits were adopted to evaluate the levels of (j) TFPI in serum, (l) TFPI in BALF, (l) MDA in BALF, and (m) NOS in BALF.

**Figure 9:** Schematic overview of the mechanism between ZNF354C, TFPI, and DNMT1 based on the findings of the study. ZNF354C interacts with TFPI and upregulates TFPI by preventing TFPI promoter methylation in OGD/R-induced HUVECs. DNMT1 reduces the interaction of TFPI and ZNF354C. Functionally, ZNF354C ameliorates LIRI by preventing TFPI methylation to upregulate TFPI.

## Data Availability

The data and study materials that support the findings of this study will be available to other researchers from the corresponding authors upon reasonable request.

## Abbreviations

I/R: Ischemia reperfusion
LIRI: Lung ischemia-reperfusion injury
ALI: Acute lung injury
PGD: Primary graft dysfunction
TFPI: Tissue factor pathway inhibitor
OGD/R: Oxygen glucose deprivation/reoxygenation
HUVECs: Human umbilical vein endothelial cells
shRNA: Short hairpin RNA
CTRL: Control
OE: Overexpression
CCK-8: Cell Counting Kit-8
FITC: Fluorescein isothiocyanate
EdU: 5-Ethynyl-2′-deoxyuridine
RT-qPCR: Real-Time Quantitative PCR
PCR: Polymerase Chain Reaction
RT: Reverse transcription
BCA: Bicinchoninic acid assay
SDS: Sodium dodecyl sulfate
PAGE: Polyacrylamide gel electrophoresis
PVDF: Polyvinylidene fluoride
GAPDH: Glyceraldehyde-3phosphate dehydrogenase
DAPI: 2-(4-Amidinophenyl)-6-indolecarbamidine dihydrochloride
MS-PCR: Methylation-specific polymerase chain reaction
ChIP: Chromatin immunoprecipitation
PBS: Phosphate-buffered saline
min: Minute
WT: Wild-type
EMSA: Electrophoretic mobility shift assay
UV: Ultraviolet ray
ELISA: Enzyme-linked immunosorbent assay
MDA: Malondialdehyde
NOS: Nitric oxide synthase
BALF: Bronchoalveolar lavage fluid
IHC: Immunohistochemistry
H&E: Hematoxylin and eosin.

## Supplementary Materials

Supplementary 1 Figure S1: quantitative analysis of ROS level. The level of ROS was tested with DCFDA/H2DCFDA-Cellular ROS Assay, and relative fluorescence intensity was counted in the corresponding groups. The experiment was repeated three times independently.

Supplementary 2 Figure S2: quantitative analysis of TFPI in IHC results. The relative intensity of TFPI was quantitatively analyzed based on the IHC results in Figure 7(f).
